The article "Automatic Identification of MALDI-TOF MS Database Using Classical Bordetella Species Isolates" was published in 2022. Journal: Comput Math Methods Med.

# Automatic Identification of MALDI-TOF MS Database Using Classical *Bordetella* Species Isolates

**DOI:** 10.1155/2022/1679951

**Published:** 2022-06-15

**Authors:** Yamin Liu, Junwen Cui, Chunhua Qie, Bei Jiang, Ying Li, Xiaoyun Zhao

**Affiliations:** ^1^Clinical School of the Second People's Hospital, Tianjin Medical University, Tianjin 300192, China; ^2^College of Basic Sciences, Tianjin Agricultural University, Tianjin 300384, China; ^3^Tianjin Institute of Hematology, Tianjin 300192, China; ^4^Department of Infectious Disease, Tianjin Second People's Hospital, Tianjin 300192, China; ^5^Chest Clinical College of Tianjin Medical University, Tianjin 300070, China; ^6^Department of Respiratory Critical Care Medicine and Sleep Center, Tianjin Chest Hospital, Tianjin 300222, China

## Abstract

**Objective:**

To evaluate and expand the automatic identification and clustering of clinical *Bordetella* species by MALDI-TOF MS.

**Methods:**

Twenty-eight field isolated strains, identified by whole-gene sequencing analysis, were analyzed by MALDI-TOF MS, and the spectra obtained were used to replenish the internal database of the manufacturer. To evaluate and expand the robustness of the database, MALDI-TOF MS identified 91 clinical isolates (except those used for implementation). A distance tree based on mass spectrometry data is constructed to confirm similarity and clusters of each clinical *Bordetella* species by using the MALDI Biotyper 3.1 software.

**Results:**

In this research, when we used the implemented Bruker Daltonics database in our laboratory, 91 clinical isolates were identified at the genus level (100%) and 93.4% were identified at the species level (85/91). We performed proteomics analysis and divided these 91 isolates into cluster I (2.2%) and cluster II (97.8%). The largest group is cluster II (*n* = 89 isolates), which has been divided into two subclusters. Trees created by analyzing the protein mass spectra of the three species of the clinical isolates reflected their classification.

**Conclusion:**

MALDI-TOF MS may present an attractive alternative to automatically confirm and cluster the fastidious bacteria difficult to culture. Extension of identification of the MALDI-TOF MS database is viably fast, more efficient, and alternative to conventional methods in confirming the classical Bordetella species. This strategy could promote the epidemiological and taxonomic research of this important pathogen.

## 1. Introduction

Pertussis disease, also known as whooping cough, is a vaccine-preventable infectious disease caused by the bacterium called *Bordetella pertussis* (Bp). Infants too young to be vaccinated or not fully vaccinated are the most severely infected groups [1, 2]. Despite the wide coverage of vaccination, the resurgence of pertussis has been observed in many countries around the world [3, 4]. There are additional members of the *Bordetella* family, such as *Bordetella parapertussis* (Bpp) and *Bordetella* bronchiseptica (Bb) (usually known as the classical *Bordetella* species), which are also related to respiratory tract infections in humans or animals.

The article "Automatic Identification of MALDI-TOF MS Database Using Classical Bordetella Species Isolates" was published in 2022. Journal: Comput Math Methods Med.

To implement effective prevention and control measures for *Bordetella pertussis*, we should be able to confirm this pathogen precisely. Bacterial culture has been considered to be the gold standard for detection of *Bordetella pertussis*. In the past years, the identification of Bp has mainly depended on a biochemical test, slide agglutination, and polymerase chain reaction (PCR) [5]. But these techniques have many shortcomings and require certain professional knowledge to accurately confirm and classify [6].

Recently, MALDI-TOF MS has become a breakthrough method for rapid, routine identification of microorganisms with excellent cost-effectiveness, high reproducibility, and reliability. The principle of this technology is to extract unique and representative spectral signals from microorganisms and establish the corresponding recognition relationship by matching the signal pattern with the pattern of the reference strain in the database. It is a rapid and reliable microbial identification and clustering technology [7, 8]. However, MALDI-TOF MS for identification and cluster analysis on *Bordetella* species has rarely been reported. The commercialized Bruker Biotyper database (DB-5989MSP) available contained *Bordetella* species with small amount of bacterial spectrum information, but the spectrum database of other brands of mass spectrometers has not included *Bordetella* species spectrum information. In order to make it possible to confirm the isolated classic *Bordetella* species more accurately in our region, we used clinical strains to evaluate and expand the capability of the MALDI Biotyper system to confirm, cluster, and analyze classical *Bordetella* species.

## 2. Materials and Methods

### 2.1. Bacterial Strains

A total of 119 *Bordetella* species isolates from infants of 0-6 months with suspected whooping cough were collected from 2018 to 2019 in the infectious center of Tianjin Second People's Hospital, China. The isolated strains were mainly from nasopharyngeal swabs or nasopharyngeal aspirates. Bacterial strains were cultured on charcoal agar (Oxoid Ltd., England) with the addition of 10% sheep blood and 40 *μ*g/ml cephalexin (*Bordetella* Selective Supplement; Oxoid Ltd.) (BORDC medium) at 37°C with 5% CO_2_ for 3-7 days and inspected regularly, as previously reported [9]. Presumptive *Bordetella* colonies with a grey morphology were measured by MALDI-TOF MS. Twenty-eight field isolated strains were identified by whole-gene sequencing analysis performed by MALDI-TOF MS, and these spectra were utilized to replenish the manufacturer internal data (Bruker Daltonik GmbH). In order to evaluate and expand the robustness of the database, MALDI-TOF MS identified 91 clinical isolates (except those used for implementation).

The article "Automatic Identification of MALDI-TOF MS Database Using Classical Bordetella Species Isolates" was published in 2022. Journal: Comput Math Methods Med.

### 2.2. Sample Preparation for MALDI Biotyper Analysis

Proteides were pretreated using the procedure of ethanol/formic acid extraction as previously described [10]. Suspended bacterial colonies in 300 *μ*l distilled water and 900 *μ*l of ethyl alcohol were vortexed for 30 seconds and then centrifuged at 10,000 × *g* for 2 minutes. Remove the supernatant, then centrifuge 2 times, remove excess ethanol, then dry at common temperature, and resuspend the precipitate in 50 *μ*l of 70% formic acid aqueous solution and 50 *μ*l in acetonitrile solution. Mix samples thoroughly at 10,000 × *g* for 2 minutes, and spot 1 *μ*l supernatant onto a 96-target polished steel plate (Bruker Daltonik). Dry at room temperature, and 1 *μ*l of HCCA (alpha-cyano-4-hydroxycinnamic acid) was dropped on the sample and waited to crystallize.

### 2.3. MALDI-TOF MS Database Expansion for *Bordetella* Species

The commercialized Bruker Biotyper database (DB-5989MSP) available already contained 10 spectra for *Bp*, 11 spectra for *Bpp*, and 9 spectra for *Bb*. This database also contained spectra for the other species of *Bordetella*, except *Bordetella ansorpii*. In order to make it possible to confirm the isolated classic *Bordetella* species more accurately in our region, we expanded the commercialize Bruker Biotyper library in our experience. Each of the 28 strains was analyzed and supplemented in the Bruker Biotyper library (DB-5989MSP) confirmed by MALDI-TOF MS and Whole-Genome Sequencing (WGS). BTS was used as an internal calibration procedure. Spot each sample at 8 locations of the target and about 24 original spectra of each strain. The spectra obtained were analyzed by using the flexAnalysis software (version 3.0, Bruker Daltonics) for “smoothing” and “baseline,” and the spectrum with intensity less than 10^4^ unitary units and singlet spectra with different peaks were selected. As described previously [11], these selected spectra were removed by using the automation function on the MALDI Biotyper software (Biotyper MSP Creation Standard Method, Bruker Daltonics), and the rest was used to reckon the reference in the main spectral profile (MSP).

For the sake of obtaining typical results, at least 20 spectra were applied to set up a singlet MSP proponent by Bruker Daltonik GmbH (Bremen, Germany). Although the automation function on MALDI Biotyper software was utilized, these remaining required spectra were used to reckon the reference in MSP. The MSP spectra were used for MALDI Biotyper database expansion and implementation.

The article "Automatic Identification of MALDI-TOF MS Database Using Classical Bordetella Species Isolates" was published in 2022. Journal: Comput Math Methods Med.

### 2.4. MALDI Biotyper Analysis

The MALDI Biotyper RTC software version 3.1 (Bruker Daltonik) was used for bacterial identification. Kations were pretreated at accelerating voltage of 20 kV, and spectra were analyzed in the positive linear mode at a mass charge ratio (*m*/*z*) of 2,000 to 20,000 Da. Adjust the laser intensity of the sample to be slightly above the ionization threshold and desorption thresholds. Each optical spectrum represents a single proteide spectrum of a bacterial strain. After automatic acquisition, the spectrum of the test bacteria, acquired through the MALDI Biotyper RTC, is transformed into a peak list. The bacterial test standard (BTS) was calibrated by using a Bruker Daltonics instrument. And the spectra were analyzed by using the Bruker Biotyper library (DB-5989MSP) and the expanded in-house MALDI-TOF MS database. 10 best matches and the corresponding matching score were shown in the result report for each sample. According to the matching MSP and the corresponding final logarithmic score, the identification results are displayed in the score table.

According to the Bruker's proprietary algorithm, this peak list is compared to the reference peaks of organism in the reference database, and a score value range from zero to three is calculated. The high score means a high degree of similarity compared with a given organism in the reference database. Briefly, 0 to 1.699 indicates that there is no reliable identification, 1.700 to 1.999 indicates a possible genus-level identification, 2.000 to 2.299 indicates a safe genus-level identification and a possible species-level identification, and 2.300 to 3.000 indicates a highly possible species-level identification [12].

### 2.5. Principle Component Analysis (PCA) of the Analyzed Genomic Strains

To compare each strain, the spectra of the 91 examined strains were loaded into the program ClinProTools for automatic recalibration. Generate classification models. Here, specific software algorithms were used, including Quick Classifier (QC)/Different Average, Supervised Neural Network (SNN), and Genetic Algorithm (GN). According to the selected algorithm, these algorithms propose the list of identification peaks of the analytical spectrum. The statistical test of the dataset was carried out on the basis of principal component analysis (PCA), and the results were exhibited in the three-dimensional score map automatically created by that software.

The article "Automatic Identification of MALDI-TOF MS Database Using Classical Bordetella Species Isolates" was published in 2022. Journal: Comput Math Methods Med.

### 2.6. Cluster Analysis

For MALDI-TOF MS cluster analysis, 91 isolated straints reference spectra, following be called MSPs (Main Spectral Profiles), independently created. Each of the extracted samples of the prepared representative strain was dropped on 8 points on the polished steel plate and then tested three times by averaging data from 240 laser shots using MALDI Biotyper software to generate 24 qualified mass spectra, which were subsequently composed of one MSP. MSPs of the strains were used to cluster the classical *Bordetella* species. Based on the values obtained from the MSPs of each strain, a tree was generated, allowing visualization of the similarities among all spectrum profiles. Use the comprehensive statistical tool MATLAB 7.1 of the Biotyper 3.1 software toolbox to process hierarchical cluster analysis and the default correlation function.

## 3. Results

### 3.1. Accuracy of Identification by MALDI-TOF MS

All 91 strains were subjected to analysis by MALDI Biotyper RTC software version 3.1, and acquired spectra were aligned to the Bruker Biotyper library (DB-5989MSP) and the implemented database. The results of the log score obtained by MALDI-TOF MS identification are shown in Table 1. According to the results of MALDI-TOF MS, classify the 91 strains as 89 *Bp*, 1 *Bpp*, and 1 *Bb* at the species level. When using the implemented Bruker Daltonics database in our laboratory, all isolated strains were confirmed at the genus level (100%) and 93.4% were confirmed at the species level (85/91). Bp strains were 89 cases. Among them, there were 60.7% (54/89) strains with the reliability score of 2.0-2.229 (accurately identified genus) before the expansion of the Bp database. There were 37.1% (33/89) strains with a score of 1.700-1.999 and only 2.2% (2/89) strains with a score > 2.300 (accurately identified species). After the expansion of the database, there were 93.3% (83/89) strains with a reliability score of >2.300 and 67.4% (6/89) strains with a score of 2.000-2.229 and no strains with a score of <2.000.

### 3.2. Principle Component Analysis (PCA) of the Analyzed Genomic Strains

The PCA software in ClinProTools was used for the analysis database in visualizing the homogeny and neterogeny of these proteide spectrum. PCA can debase the diverse complex datasets based on different statistical tests. The reduced datasets, which are called PCs (principle components), can be exhibited in a plot diagram. A total of 91 individual protein spectra of the clinical *Bordetella* species are exhibited in a three-dimensional PCA in Figure 1. Each plot diagram means an exhibited proteide spectrum. These colors stand for the counted cluster members, where each point delegates a measured protein mass spectrum profile of each sample.

The article "Automatic Identification of MALDI-TOF MS Database Using Classical Bordetella Species Isolates" was published in 2022. Journal: Comput Math Methods Med.

### 3.3. Cluster Analysis

Create an MSP tree (Figure 2) to visually compare the relationships between each mass spectrum got from these 91 isolates. For a preset bacterial strain, use the rigorous data processing algorithms on MALDI Biotyper 3.1 software for creating the spectrum profile for each sample. The mass spectrum patterns were used to study the diverse technicality for confirming 91 different isolated strains. In the MSP tree view, the relative distance among isolates was exhibited as an arbitrary unit. Zero means complete similarity, and 1000 means complete dissimilarity. The willful distance level of 500 was selected for cluster evaluation of isolated strains. Our cluster analysis of all MSPs divided these *Bordetella* isolates into two clusters: cluster I, which contained 2 (2.2%) isolates, and cluster II, which contained 89 (97.8%) isolates. Cluster II, as the largest group, has been divided into two subclusters.  Figure 3 shows that all peaks are exhibited for the 89 *Bp* (black), 1 *Bpp* (red), and 1 *Bb* (green), and ion intensities, peak positions, and peak frequencies derived from the 91 isolates, representative strain of the two clusters, are the function of the *m*/*z* values. Total peaks for the 91 isolates were produced by flexAnalysis 3.3 software. Representative strains of mass spectrometric profiles of *Bp* and *Bpp* isolates are shown in Figure 4.

## 4. Discussion

*Bordetella pertussis*, as an exclusive human pathogen, can cause pertussis disease, a contagious infection in the human respiratory tract [13]. Pertussis continues to be an important cause of morbidity worldwide and of mortality in infants, especially under 6 months [14, 15]. The symptoms in clinic vary with age, former infection with *B. pertussis*, and vaccinated status. In those with incomplete immunity, pertussis can develop in atypical clinical forms and is difficult to be diagnosed [16]). The clinical manifestations in newborns may be severe. Most infants have typical spasmodic paroxysmal cough that lasts for more than two months [17]. Pertussis in children under 1 year of age is particularly difficult to diagnose in winter because of other pathogens such as influenza or respiratory syncytial virus (RSV) epidemics [18, 19].

In clinic practice, diagnosis is often given without any microbiological basis leading to a possibility that cannot initiate treatment early and prevent complications primitively. Confirming *Bordetella pertussis* in the laboratory is difficult and contributes to underreporting of the disease [20]. The operation method of the biochemical test is cumbersome and time-consuming, and slide agglutination requires a special antigen reagent, and both the false positive and false negative rates are high, also needing a professional operator [6]. There is an urgent need for a reliable device for rapid diagnosis of pertussis. By MALDI-TOF MS entering the clinical laboratory, the identification of this nutrient-critical and slow-growing bacterium has been improved [21]. In the past few years, MALDI-TOF MS has gradually been extensively used for quickly confirming and typing a variety of bacteria and fungi in the clinical microbiological laboratory [22–24]. This MALDI-TOF MS identification is mainly based on the differences of whole proteins, especially ribosomal proteins, which are automatically matched with the database. Furthermore, the technology will be automated, has high throughput, and is suitable for a wide range of common and esoteric bacteria and fungi [25, 26]. Due to the large regional differences of Bp strains, the existing mass spectrometry library cannot meet the needs of accurate identification of local epidemic strains.

The article "Automatic Identification of MALDI-TOF MS Database Using Classical Bordetella Species Isolates" was published in 2022. Journal: Comput Math Methods Med.

In this work, we analyzed and supplemented 28 strains in the Bruker Biotyper library (DB-5989MSP), which had been confirmed by Whole-Genome Sequencing (WGS). Then, we evaluated the performance of MALDI-TOF MS to rapidly detect the *Bordetella* species, using 91 previously characterized isolates, in order to consider it as an alternative tool for confirming the fastidious bacteria within minutes instead of hours and days. However, when using the implemented Bruker Daltonics database in our laboratory, all of isolates were confirmed correctly at the genus level (100%) and 93.4% (85/91) were confirmed at the species level. Bp species was confirmed correctly at the genus level (100%), and 93.3% (83/89) was confirmed at the species level. These results show that the accurate identification of bacteria depends on the quality of the database. Thence, the Biotyper database needs to be expanded by additional more spectra to create one representative database, to promote the matching score and achieve highly precise species-level identification. The implementation of the database reinforced the scores of identification of the classical *Bordetella* species. This will be very important for future applications in clinics.

A further main objective of our study was to assess the capability MALDI-TOF for the clustering of the *Bordetella* species. MALDI-TOF has been reported to be successfully applied for cluster analysis of many pathogens [27, 28]. Based on the data obtained from the paired comparisons of different spectra, a tree view was generated, which allows visualization of the similarity among all the spectral profiles. Our cluster analysis of all major spectra classified these *Bordetella* species to two clusters: cluster I, which contained 2 isolates (2.2%), and cluster II, which contained 89 isolates (97.8%). Except for the bacterial culture time, only 30 minutes were necessary to carry out the entire identification process, starting from the picking of the single colony and ending in analysis by MALDI-TOF MS. The MSP dendrogram is considered a reliable tool for illustrating the capability of MALDI-TOF MS to visualize the degree of similarities and differences between species when more isolates are considered [29, 30]. The manifestation of MALDI-TOF for cluster analysis was evaluated as one extended and complementary typing method, especially for the screening purpose. We expanded the sensitive culture method by screening with MALDI-TOF MS for the identification and clustering of the classical *Bordetella* species. Automatic identification and clinical analysis may be achieved by deep learning or predictive control techniques [31] and may be useful in the performance evaluation of analytical procedures in the future.

The article "Automatic Identification of MALDI-TOF MS Database Using Classical Bordetella Species Isolates" was published in 2022. Journal: Comput Math Methods Med.

## 5. Conclusion

In summary, our study strongly indicates that using classical *Bordetella* species isolates can expand automatic identification of the MALDI-TOF MS database. Extension of identification of the MALDI-TOF MS database is viably fast, more efficient, and alternative to conventional methods and may aid in the surveillance of regional strains of the classical *Bordetella* species. It may present an attractive alternative to confirm and cluster the fastidious bacteria difficult to culture. This strategy could automatically facilitate the epidemiological and taxonomic research of the important pathogen.

## Figures and Tables

**Figure 1:** Principle Component Analysis (PCA) of the analyzed genomic strains. Datasets of the genomospecies *Bp*, *Bpp*, and *Bb* were analyzed using the ClinProTools software.

**Figure 2:** The MSP tree of the 91 isolated strains, which was created based on mass signal patterns by using the MALDI Biotyper 3.1 software. Clusters I and II are exhibited. The distance level showing the overall similarity between 91 isolates was standardized relative to the maximum value of 1000.

**Figure 3:** The mass spectrum of the *Bordetella* species isolates created by using flexAnalysis 3.3 software shows that ionic strength (*y*-axis) is a function of the mass charge ratio (*m*/*z*, *x*-axis). All peaks are exhibited for the 89 *Bp* (black), 1 *Bpp* (red), and 1 *Bb* (green).

The article "Automatic Identification of MALDI-TOF MS Database Using Classical Bordetella Species Isolates" was published in 2022. Journal: Comput Math Methods Med.

**Figure 4:** Representative strain of mass spectrometric profiles of *Bp*, *Bpp*, and *Bb* isolates.

**Table 1:** The identification scores of 91 isolates of *Bordetella* species analyzed using the Bruker Daltonics database and our new database.

Genomospecies	MALDI-TOF identification using DB-5989MSP				MALDI-TOF identification using the implemented database			
	>2.300	2.000-2.299	1.700-1.999	Total	>2.300	2.000-2.299	1.700-1.999	Total
*B. pertussis*	2	54	33	89	83	6	0	89
*B. parapertussis*	0	1	0	1	1	0	0	1
*B. bronchiseptica*	0	1	0	1	1	0	0	1

Scores of 0 to 3 (log10) were assigned according to spectral peak patterns as follows: >2.300, secure species identification; 2.000 to 2.299, secure genus identification; 1.700 to 1.999, probable genus identification; and <1.700, no reliable identification.

## Data Availability

Data are available on request from the authors due to privacy/ethical restrictions.
